# Effect of GuiXiong Xiaoyi Wan in Treatment of Endometriosis on Rats

**DOI:** 10.1155/2015/208514

**Published:** 2015-01-27

**Authors:** Zhixing Jin, Li Wang, Zhiling Zhu

**Affiliations:** ^1^Shanghai Medical College of Fudan University, Shanghai 200011, China; ^2^Obstetrics and Gynecology Hospital of Fudan University, Shanghai 200011, China

## Abstract

*Objective*. To evaluate the effect of GuiXiong Xiaoyi Wan (GXXYW) on the development of endometriosis in a rat model. *Methods*. Sprague-Dawley rats with surgically induced endometriosis were randomly treated with low-dose GXXYW, high-dose GXXYW, or vehicle (negative control) for 28 days. Immunohistochemistry was used to assess cell proliferation in the lesions. The terminal deoxynucleotidyl transferase- (TdT-) mediated dUTP biotin nick end labelling (TUNEL) method was performed to analyse the apoptosis induced by GuiXiong Xiaoyi Wan. The percentages of CD3+ lymphocytes, CD4+ lymphocytes, and CD8+ lymphocytes in the spleens of the rats were evaluated using flow cytometric analysis. *Results*. Treatment with GXXYW significantly decreased the lesion size, inhibited cell proliferation, and induced apoptosis in endometriotic tissue. The spleens of GXXYW-treated rats also demonstrated a significant increase in the percentage of CD4+ lymphocytes and a significant decrease in the percentage of CD8+ lymphocytes. *Conclusions*. These results suggest that, in a rat model, GXXYW may be effective in the suppression of the growth of endometriosis, possibly through the inhibition of cell proliferation, the induction of apoptosis of endometriotic cells, and the regulation of the immune system.

## 1. Introduction

Endometriosis is a hormone-dependent benign disease that affects at least 10% of reproductive-aged women and is characterized by the presence of a functional endometrium outside of the uterine cavity [1]. Although it is actively researched by scientists all over the world, the pathogenesis of endometriosis is still unknown. By far, the most widely accepted hypothesis that explains the pathogenesis of endometriosis is retrograde menstruation, which was proposed by Sampson in 1927 [2].

Recently, many studies have indicated the important role of immunology in the pathogenesis of endometriosis [3]. Particularly, in cell-mediated immune responses, T lymphocytes play essential roles in the response to autologous endometrium, such as the determination to either accept or reject survival, implantation, and proliferation of endometrial and endometriotic cells [4]. Numerous studies have shown aberrant changes in T lymphocytes in women with endometriosis [5]. T lymphocytes originate from pluripotent stem cells and develop into two major subpopulations called helper T-cells or CD4+ T cells and cytotoxic T-cells, which are characterized by the expression of the glycoprotein CD8. Classic studies that examined the CD4 : CD8 ratio showed that the ratio was decreased in endometriotic peritoneal fluid (PF) [6], which suggested that a diminished cellular-mediated immune response could facilitate the ectopic implantation of the translocated endometrial cells [7].

Currently, surgery and medicine are the standard therapeutic options for endometriosis. Although endometriotic lesions can be removed during surgery, this rarely eliminates all of the lesions, and postoperational relapse is unavoidable [8]. In Western medicine, pseudopregnancy therapy such as oral contraceptives and pseudomenopause therapy such as gonadotropin-releasing hormone-analogs (GnRH-a) are often effective in the short-term treatment of this disease; however, the consequent side effects limit the use of these therapies for a longer duration [9].

In Chinese medicine, endometriosis is considered a syndrome caused by blood stasis [10]. Many recent studies have illustrated that Chinese medicine (CM) therapy has achieved good results in the alleviation of pain, the promotion of fertility, and the prevention of relapse [11]. In addition, CM allows for individualized therapy according to each patient's special requirements. The formula, or* fufang*, contains a combination of different types of plants to improve clinical efficacy. GuiXiong Xiaoyi Wan (GXXYW), a Chinese medicinal formula for endometriosis, is prescribed by practitioners based on their clinical experience. In our clinical practice, we have found that GXXYW can alleviate endometriosis-related symptoms. However, the mechanisms of how it affects endometriosis remain unknown.

In our study of a rat model of endometriosis, we examined the influence of GXXYW on cell proliferation and apoptosis of endometriotic cells, and the percentages of CD3+ lymphocytes, CD4+ lymphocytes, and CD8+ lymphocytes in the spleens of rats.

## 2. Materials and Methods

### 2.1. Preparation of Formula and Animals

The species of the herbs that comprise GXXYW are listed in Table 1.

All of the medicinal plants consist of formulas that were provided by the Obstetrics and Gynecology Hospital of Fudan University on the Integration of Chinese and Western Medicine (Shanghai, China). The plants, with the exception of* Draconis Sanguis*, which cake under high-temperature conditions, were homogenized with a Waring blender and decocted in double-distilled water to 100°C for 1.5 h. Then, the decoction was filtered and concentrated by heating. Finally, the* Draconis Sanguis* powder was added and the solution was mixed.

Fifty mature, female, nonpregnant Sprague-Dawley rats that weighted between 200 g and 220 g were obtained from the Laboratory Animal Center of the Shanghai Institutes of Biological Sciences. They were caged in a controlled environment at 22°C with 12 h light/dark cycles. All food and water were sterilized and provided* ad libitum*. All rats were allowed to have 7 days to acclimate to the environment before the experiments were performed. All experiments in this study were conducted according to the guidelines of the National Research Council's Guide for the Care and Use of Laboratory Animals and were approved by the Institutional Experimental Animals Review Board of Shanghai Academy of Traditional Chinese Medicine [12].

### 2.2. The Rat Model of Endometriosis and Animal Treatment

Fifty rats were divided into two groups: a group of 10 rats served as the sham-operated controls, and the remaining 40 rats were used for the rat model of endometriosis. Briefly, animals were anesthetized with an intraperitoneal administration of 10% chloral hydrate (m/v) at 0.7 mL/200 g body weight. The rats used for this model of endometriosis underwent laparotomy by midventral incision to expose the uterus. The right uterine horn was removed and placed in a Petri dish containing warmed phosphate-buffered saline (PBS). The uterine horn, which was opened longitudinally and sectioned into a 5 × 5 mm piece, was transplanted onto the outer surface of the right abdominal wall with the endometrium facing the peritoneal cavity. A 6-0 nylon suture line was used to attach the graft. The remaining ten rats that formed the sham-operated group were subjected to unilateral hemihysterectomy without the autotransplantation of the uterine tissue. The midventral abdominal incision was closed with 3-0 sutures. After surgery, penicillin was injected for 3 days at 400 000 units per rat. Two days after surgery, they were injected with 0.1 mg/kg/day of estradiol every 4 days, for a total of three times, which can promote the growth of ectopic endometrium [13].

After a recovery period of 28 days, the 40 rats that were used for the rat model of endometriosis underwent a second exploratory laparotomy to examine if models of experimental endometriosis have been successfully established, which was determined by observation of red/brown color and cystic formation on implant surfaces [14], then the volume of the endometrial implants was measured to make sure all of the rats showed a similar size of endometriotic lesions. Thirty rats, in which experimental endometriosis was successfully established and showed a similar size of endometriotic lesions, were randomly divided into three groups as follows: the control group, the GXXYW low-dose group, and the GXXYW high-dose group. Each group consisted of 10 rats. The rats in the GXXYW low-dose and high-dose groups were administered, by oral gavage for 28 days, GXXYW at 13 g/kg/day and 26 g/kg/day, respectively. The low dose was calculated using the formula of dose translation among different species based on body surface area [15]. The dose of GXXYW for women was 116 g, and the body weight of women was taken as 55 kg. So, the expected dose for rats was 13 g/kg, which was similar to that for women. To further explore whether the effect of GXXYW was dose dependent and to avoid the possibility that rats may have higher tolerance for GXXYW than women, we also took the 2-fold dose. The rats in the sham-operated group and the control group received an equal volume of double-distilled water for 28 days.

### 2.3. Specimen Collection

After treatment for 28 days, the rats were sacrificed by cervical dislocation. Each lesion (normal endometrium for the sham-operation group) was dissected, immediately fixed in 4% paraformaldehyde solution, and then embedded in paraffin for immunohistochemical study. The spleens of the rats in each group were washed with physiologic saline for the isolation of T lymphocytes.

### 2.4. Immunohistochemistry

Each paraffin-embedded tissue block was subjected to serial 3 mm sectioning for haematoxylin and eosin staining for the pathologic confirmation and subsequent immunohistochemical staining for PCNA (clone PC10, Cell Signaling Technology, Denver, CO, USA). The slices were subjected to antigen retrieval with citric acid buffer (pH 6.0) and were then incubated with diluted primary antibody (1 : 2000) overnight at 4°C. After washing in PBS (pH 7.4) 3 times for 15 min, the sections were incubated with diluted (1 : 50) secondary antibody for 60 min. Subsequently, the slides were washed again in PBS and incubated with 0.01% 3,3-diaminobenzidine tetrahydrochloride (DAB) for approximately 2 min. Sections were then washed thoroughly in PBS 3 times for 5 min each, counterstained in haematoxylin for 20 s, dehydrated in absolute alcohol, cleared in xylene, and mounted in synthetic resin for microscopic examination. The number of cells that expressed PCNA per 100 total cells was established by two independent observers using a standard light microscope [16]. The total number of cells in ten representative fields was counted. Any nuclear staining was regarded as positive.

### 2.5. TUNEL Assay

Paraffin sections were washed in xylene twice for 10 min each and hydrated with 100% ethanol, 95% ethanol, and 75% ethanol for 5 min each. They were then washed twice in PBS, then incubated with 0.1% Triton X-100 in 0.1% sodium citrate for 8 min and rinsed in two changes of PBS for 5 min each. A total of 25 *μ*L of TUNEL reaction mixture was added to each sample, which was then covered and incubated for 60 min at 37°C in a humidified atmosphere in the dark. The slides were rinsed with PBS 3 times for 10 min each followed by incubation with DAPI for 2 min at room temperature to stain the nuclei. The slides were rinsed in PBS 3 times and placed on a coverslip with antifade mounting medium (Life Technologies, Waltham, MA, USA).

### 2.6. Flow Cytometric Analysis of T-Cells in the Spleen

The splenic tissue was minced using a tissue grinder and rinsed with PBS (pH = 7.4). The suspension was isolated by covering it with rat lymphocyte separation medium (Dakewe, Shanghai, China) and by centrifugation at 2000 rpm for 30 min. The isolated mononuclear cells were removed to another centrifuge tube and washed twice with PBS, and then the cell concentration was adjusted to 10^6^ cells/100 *μ*L. The mononuclear cells that were isolated by the rat lymphocyte separation medium were incubated with fluorescently labelled antibodies CD3 (BioLegend, San Diego, CA, USA), CD4 (BioLegend, San Diego, CA, USA), and CD8a (BioLegend, San Diego, CA, USA) at 4°C for 30 min. The cells were washed twice in PBS and resuspended in 500 *μ*L of PBS. Cell counts were performed on a FACSCalibur machine (Becton Dickinson, Franklin Lakes, NJ, USA) and the data were collected for 10,000 events/sample using CELLQuest (Franklin Lakes, NJ, USA).

### 2.7. Statistical Analysis

All statistical analyses were performed using the software SPSS 16.0 for Windows (Chicago, IL, USA). Statistical comparisons were made by Kruskal-Wallis test. Differences between groups were considered statistically significant at *P* < 0.05.

## 3. Results

### 3.1. Treatment with GXXYW Reduces the Volume of the Lesion

Experimental endometriosis was successfully established in 30 rats using the protocol described above. These rats then underwent a second exploratory laparotomy for the examination of the endometrial implants and make sure all of the rats showed a similar endometriosis stage. After the 28-day treatment with GXXYW, the longest lengths and perpendicular widths of the lesions were measured by a vernier calliper. The volume of the endometriotic lesion was calculated by 0.52  ×  width^2^  ×  length [17]. A comparison of the GXXYW-treated groups and the control group demonstrated a statistically significant reduction in the lesion size after the treatment, and, as the dose increased, the volume of the lesion size was further reduced (Figure 1 and Table 2).

### 3.2. Treatment with GXXYW Inhibits Cell Proliferation

The histopathologic findings showed typical endometrial histomorphology in the lesions (Figure 2(a)). Cell proliferation was evaluated by immunohistochemistry for the presence of PCNA. As illustrated in Figure 2(b) and Table 3, compared with the rats in the sham-operation group, the number of PCNA-positive cells of the lesions from the control rats was increased significantly. Treatment with GXXYW caused a decrease in cell proliferation in the lesions compared with the control group, which was unrelated to the dose.

### 3.3. GXXYW Induces Apoptosis in Ectopic Endometrial Tissue

As shown in Figure 3, all endometriotic tissues were scattered among the TUNEL-labelled cells and positive signals were localized in the nucleus, as indicated by green fluorescence. Compared with the control group, endometrial tissue that was treated with different doses of GXXYW contained an increased number of positive cells. The number of positive cells increased along with increasing doses of GXXYW, which suggests that GXXYW can achieve an antiproliferative effect, possibly via the induction of apoptosis in endometriotic tissue.

### 3.4. Assay of the Percentage of T Lymphocytes in the Spleen

After treatment for 28 days, as it is shown in Figure 4 and Table 4, a comparison of the rats in the control group shows a statistically significant increase in the percentage of CD4+ lymphocytes and a decrease in the percentage of CD8+ lymphocytes in the spleens of rats in both groups that were treated with GXXYW; these changes were not related to the dose. The differences in the number of CD3+ lymphocytes in the spleens of rats of the different groups were not statistically significant.

## 4. Discussion

In China, traditional herbal preparations still account for 30–50% of the total medicinal consumption [18]. Due to better efficiency and fewer side effects, traditional medicine, also called complementary and alternative medicine (CAM), is popular in all regions of the developing world, and its use is spreading rapidly in developed countries [19]. In recent years, medicinal herbs have become popular for the management of endometriosis-associated symptoms [20]. GXXYW treatment is designed by practitioners based on their clinical experience for patients with endometriosis to resolve blood stasis. In the current study, we examined the therapeutic potential of GXXYW, determined its ability to reduce ectopic growth, and explored the possible mechanism of action in an animal model, which can provide theoretical foundation for endometriosis treatment and let us know more about pathogenesis of this disease.

Our studies of a rat model of endometriosis demonstrated that a physiological dose (which is 10 times as many as the amounts administered to humans) of GXXYW given for 28 days caused a significant reduction in the volume of the lesion size, and, as the dose increased, the lesion became smaller. It is widely accepted that apoptosis, cell proliferation, and the cell-mediated immune response contribute to the growth of endometriotic lesions [21]. Therefore, in our research, we used a TUNEL assay to examine the occurrence of apoptosis in rat endometrial cells and IHC to determine the distribution of PCNA within the lesions, which indicates cell proliferation. We found that treatment with GXXYW diminished cell proliferation and induced apoptosis in endometriotic lesions.

T lymphocytes play essential roles in the pathogenesis of endometriosis [22]. A decrease in the CD4 : CD8 ratio was observed in patients with endometriosis, which is an indication of the inhibition of the cell-mediated immune response [23]. Our present work showed that treatment with GXXYW can increase the CD4 : CD8 ratio, which suggests that it can enhance the cell-mediated immune response within patients that would result in the removal of ectopic cells.

Compared with traditional Chinese formulas that have been mostly reported, GXXYW reduced the volume of lesion size as much as Guizhi Fuling Capsule [13], which is much more than other formulas, such as Wenshen Xiaozheng Tang [24] and Sanjie Zhentong Capsule [25], and also showed a significantly improvement of cell-mediated immune response. However, there are some limitations of our study. Although biological behaviours of autologous endometrial explants were similar to human lesions in vivo, it may be more persuasive to evaluate the effects of GXXYW in human in vivo or in vitro. Another limitation of our study was that we only assessed the effects of GXXYW using different doses and did not compare with traditional western and Chinese medicine that have already been used clinically. In our research, we only find some aspects that GXXYW may influence, so future studies should be evaluated in other fields, such as angiogenesis and inflammation.

## 5. Conclusions

In summary, the present study has shown that GXXYW significantly reduced the size of the endometrial explants in this rat model, which may be caused by the inhibition of cell proliferation, an induction in apoptosis, or the regulation of the cell-mediated immune response.

## Figures and Tables

**Figure 1:** The volume of ectopic endometrial tissue after the treatment with different doses of the GXXYW via oral gavage. (a) Comparison of the volume of the lesion size in each group after 28 days of treatment; (b) Box plot showing endometrial volumes of different groups. Rats in the control group received distilled water only; rats in the low-dose group were administered GXXYW 13 g/kg/day; rats in the high-dose group were administered GXXYW 26 g/kg/day.

**Figure 2:** Effect of GXXYW on cell proliferation in endometriotic lesions. Cell proliferation was evaluated by immunohistochemistry for the expression of proliferating cell nuclear antigen (PCNA). (a) Comparison of the percentage of PCNA+ cells in the different dose groups after 28 days of treatment; 400x Magnification. (b) Box plot showing the percentage of PCNA+ cells. Control group received distilled water only; low dose, GXXYW low-dose group; high dose, GXXYW high-dose group.

**Figure 3:** TUNEL assay of ectopic endometrial tissue in the different groups (200x magnification).

**Figure 4:** Box plots showing treatment-related enhancement of a cell-mediated immune response in the spleens of experimental rats. Splenocytes were isolated and analysed by flow cytometry for the expression of CD3+, CD4+, and CD8+ cells. (a) Box plot showing the percentage of CD3+ T cells in gate; (b) Box plot showing the percentage of CD4+ T cells in gate; (c) Box plot showing the percentage of CD8+ T cells in gate; (d) Box plot showing the ratio of CD4+ T cells/CD8+ T cells. Rats in the control group and sham group received distilled water only; rats in the low-dose group were administered GXXYW 13 g/kg/day; rats in the high-dose group were administered GXXYW 26 g/kg/day.

**Table 1:** The composition of GuiXiong Xiaoyi Wan.

Scientific name	Chinese name	Medicinal parts	Origin	Grams	%
*Angelica sinensis *	Danggui	Root	Shanxi, China	10	8
*Ligusticum wallichii *	Chuanxiong	Tuber	Sichuan, China	6	5
*Radix Astragali preparata *	Zhihuangqi	Root	Gansu, China	10	8
*Salvia miltiorrhiza *	Danshen	Root	Shandong, China	10	8
*Scalding leech *	Tangshuizhi	Whole body	Anhui, China	3	3
*Radix Paeoniae Rubra *	Chishao	Root	Neimenggu, China	10	8
*Cynanchum paniculatum *	Xuchangqing	Root	Anhui, China	10	8
*Spina gleditsiae *	Zaojiaoci	Calthrop	Jiangxi, China	6	5
*Herba epimedii *	Yinyanghuo	Overground part	Shanxi, China	10	8
*Semen persicae *	Taoren	Seed	Anhui, China	10	8
*Ground beetle *	Tubiechong	Female imago	Shandong, China	10	8
*Vinegar attached rhizoma cyperi *	Cuxiangfu	Tuber	Shandong, China	10	8
*Vinegar attached rhizoma corydalis *	Cuyanhusuo	Tuber	Zhejiang, China	10	8
*Draconis Sanguis *	Xuejie	Resin	Hainan, China	1	1

Total amount				116	100

**Table 2:** Volume of lesion after GuiXiong Xiaoyi Wan treatment.

Variable	Median (mm^3^)	Percentiles (P_25_~P_75_)
Control	97.71	86.99~111.1
Low-dose GXXYW	66.11^*^	23.47~91.54
High-dose GXXYW	28.29^*^	7.465~40.68

^*^Mean *P* < 0.05, when compared with control group.

**Table 3:** Percentage of PCNA+ cells in endometriotic lesions showingeffect of GXXYW on cell proliferation.

Variable	Median (%)	Percentiles (P_25_~P_75_)
Sham	20^*^	16.25~23.75
Control	75	65.00~82.50
Low-dose GXXYW	22.5^*^	10.00~30.00
High-dose GXXYW	20^*^	10.00~30.00

^*^Mean *P* < 0.05, when compared with control group.

**Table 4:** Treatment-related enhancement of a cell-mediated immune response in the spleens of experimental rats.

Variable	Percentage of CD3+ T cell in gate		Percentage of CD4+ T cell in gate		Percentage of CD8+ T cell in gate		CD4/CD8 Ratio	
	Median (%)	P_25_ ~P_75_	Median (%)	P_25_ ~P_75_	Median (%)	P_25_ ~P_75_	Median (%)	P_25_ ~P_75_
Sham	43.37	38.62~50.63	57.04	56.72~59.17	33.83	31.66~35.50	1.690	1.606~1.870
Control	36.62	32.03~42.88	57.11	56.81~58.22	35.09	30.47~37.82	1.628	1.518~1.899
Low-dose	40.13	29.27~45.59	64.00^*^	54.26~71.09	25.05^*^	19.28~28.78	2.560^*^	1.894~3.798
High-dose	42.16	39.50~46.68	64.26^*^	61.82~68.83	22.50^*^	19.13~23.80	2.955^*^	2.610~3.602

^*^Mean *P* < 0.05, when compared with control group.
